This article has been retracted.

# Physical Exercise and Patients with Chronic Renal Failure: A Meta-Analysis

**DOI:** 10.1155/2017/7191826

**Published:** 2017-02-20

**Authors:** Zhenzhen Qiu, Kai Zheng, Haoxiang Zhang, Ji Feng, Lizhi Wang, Hao Zhou

**Affiliations:** ^1^Minjiang University, Fuzhou, Fujian, China; ^2^Department of Urology, Fuzhou General Hospital, Fuzhou, Fujian, China; ^3^Department of Gastroenterology, General Hospital of Tibet Military Region, Lhasa, Tibet, China; ^4^Department of Gastroenterology, General Hospital of Shenyang Military Region, Shenyang, Liaoning, China; ^5^Department of Chronic Infectious Disease Prevention and Control, Hongkou District Center for Disease Control and Prevention, Shanghai, China; ^6^Department of Urology, People's Hospital Affiliated to Fujian University of Traditional Chinese Medicine (The People's Hospital of Fujian Province), No. 602, Middle Road 817, Fuzhou, Fujian, China

## Abstract

Chronic renal failure is a severe clinical problem which has some significant socioeconomic impact worldwide and hemodialysis is an important way to maintain patients' health state, but it seems difficult to get better in short time. Considering these, the aim in our research is to update and evaluate the effects of exercise on the health of patients with chronic renal failure. The databases were used to search for the relevant studies in English or Chinese. And the association between physical exercise and health state of patients with chronic renal failure has been investigated. Random-effect model was used to compare the physical function and capacity in exercise and control groups. Exercise is helpful in ameliorating the situation of blood pressure in patients with renal failure and significantly reduces VO_2_ in patients with renal failure. The results of subgroup analyses show that, in the age >50, physical activity can significantly reduce blood pressure in patients with renal failure. The activity program containing warm-up, strength, and aerobic exercises has benefits in blood pressure among sick people and improves their maximal oxygen consumption level. These can help patients in physical function and aerobic capacity and may give them further benefits.

## 1. Introduction

Renal failure is characterized with the loss of its function and results in the accumulation of metabolites in blood [1–6]. As a result, the balance of fluids and electrolytes in the body gets disturbed, thereby causing serious health problems [7–10]. A gradual loss of kidney function over a period of several years is termed as chronic kidney disease (CKD) or chronic kidney failure [11–14]. Symptoms are usually very mild and could go unnoticed for a long time. More often than not, the symptoms are noticed when it is too late, and in a majority of cases very little can be done to reverse the situation [15–18].

In the general people, the physical activity is related to improved physical capacity and further helping in the control of chronic diseases, including chronic kidney disease. It is reported that physical fitness level of hemodialysis patients tends to improve their function levels; physical activity is an important nursing intervention for patients with hemodialysis in improving their physical performances [14, 15].

Several kinds of exercise interventions containing strength training and aerobic exercise were studied [5–8, 10]. The exercise program is usually implemented twice or three times per week, and for the participation time it is about 1 hour. The period ranges from 3 months to 1 year.

Several published randomized controlled trials (RCT) studies about the effect of exercise on patients with renal failure have shown inconsistent results [12, 14–16]. As far as we know, the previous reviews suggested physical activity can improve the health situation in renal failure patients. However, there still exist some reports that physical exercise is a risk factor for patients with renal failure. Therefore, an updated meta-analysis to assess the effects of exercise on patients with renal failure is imperative.

## 2. Materials and Methods

### 2.1. Search Strategy and Study Selection

The literature search was conducted in July 2015 among multiple databases including PubMed, EMBASE, Cochrane Library, and China Journal Full-Text Database, from January 1975 to January 2015 (Figure 1). There were two researchers carrying out a comprehensive literature search independently. The following search terms were used:

(1) “renal failure” OR “kidney failure” OR “acute renal failure” OR “chronic renal failure” OR “ARF” OR “CRF” and (2) “exercise” OR “sports” OR “activity” OR “movement”. These search keywords were assembled to seek for the articles using the Boolean operator “and” without restriction. Besides, the references cited in these papers were used to complete the search.

To be qualified for inclusion in this article, researches used the following inclusion criteria: (1) the study was RCT study; (2) it investigated the correlation between exercise and renal failure; (3) these studies must be conducted on adults; (4) the population in researches should be in dialysis; (5) full text is available. Studies were excluded if they were the following: animal studies, abstracts, review articles, case reports, letters, editorials, comments, and conference proceedings. The number of studies excluded was 633, in which there were 251 animal studies, 37 abstracts, 28 review articles, 116 case reports, 36 letters, 42 editorials, 53 comments, and 70 conference proceedings. Finally, there were 9 articles selected in this meta-analysis [19–28].

### 2.2. Data Abstraction and Quality Assessment

Two reviewers independently read the full text of the manuscripts and extracted the following data from each eligible research: first author's name, country of origin, publication year, sampling size, study period, method of ascertainment of exercise and drinking, and method of ascertainment of adult renal failure.

### 2.3. Statistical Analysis

Review Manager (Version 5.0, The Cochrane Collaboration, 2011) was used to estimate the effects of the outcomes among selected reports. Continuous variables are represented by mean and standard deviation, with heterogeneity across studies using *I*^2^ statistic (a quantitative measure of inconsistency across studies). Studies with an *I*^2^ of 25% to 50% were considered low heterogeneity, *I*^2^ of 50% to 75% was considered moderate heterogeneity, and *I*^2^ > 75% was considered high heterogeneity. If *I*^2^ > 50%, potential sources of heterogeneity were tested by sensitivity analysis conducted by eliding one study in each turn and investigating the influence of a single study on the combined estimate. A subgroup analysis was implemented based on different age ranges. Furthermore, when heterogeneity was observed, a random-effect model was adopted, and while it was absent, the fixed-effect model was utilized. Funnel plots were used to examine the potential publication bias.

In addition, sensitivity analysis was conducted to test the robustness. We examine whether the quality of reports could influence the results of this analysis. After that, subgroup analysis was carried out according to different criteria such as geographical region and source of control and risk factor.

## 3. Results

### 3.1. Search Results

The initial search found 957 related publications, in which 315 were excluded for duplication. After the screening based on the titles and abstracts, 44 articles remained. Then, 35 researches were excluded because of type of article and insufficient data. In the end, 9 RCT studies were selected for this meta-analysis, in which 8 were published in English and 1 was published in Chinese.

### 3.2. Study Characteristics

The main characteristics of the selected researches are shown in Table 1. These articles were published between 1999 and 2014. All the studies were performed in different countries. Sampling size ranged from 15 to 56. The mean age was between 22.12 and 60.8. Cases in all selected studies were confirmed based on medical records or pathological findings. The data about matching were extracted from all of the included studies.

### 3.3. Meta-Analysis of Outcome Measures

#### 3.3.1. Patients' Blood Pressure

All the studies reported that physical activity is associated with the state of health. The aggregated results suggested that exercise is helpful in improving the situation of blood pressure in patients with renal failure (MD = −4.46, 95% CI [−9.11, −0.01], *P* = 0.06, *P* for heterogeneity < 0.0001, and *I*^2^ = 77%) (Figure 2).

#### 3.3.2. Patients' Maximal Oxygen Consumption

Sports can influence maximal oxygen consumption (VO2) which was supported in the included studies. The combined results demonstrated that exercise is associated with improving the situation of VO2max in renal failure patients (MD = −1.36, 95% CI [−2.06, −0.65], *P* = 0.0002, *P* for heterogeneity = 0.49, and *I*^2^ = 0%) (Figure 3).

### 3.4. Subgroup Analyses

#### 3.4.1. Patients' Blood Pressure

Subgroup analyses were performed according to age: >50 yrs, 40–50 yrs, and 20–40 yrs. In the age >50, physical activity can significantly reduce blood pressure in patients with renal failure (MD = −5.23, 95% CI [−8.13, −2.33], *P* = 0.0004, *P* for heterogeneity < 0.0001, and *I*^2^ = 86%); in the age between 40 and 50, exercise can also significantly reduce blood pressure in patients with renal failure (MD = −6.07, 95% CI [−10.37, −1.78], *P* = 0.006, *P* for heterogeneity = 0.90, and *I*^2^ = 0%); in the age between 20 and 40, the effects of sports on blood pressure among kidney failure patients is insignificant (MD = −1.25, 95% CI [−4.24, 1.74], *P* = 0.41, *P* for heterogeneity = 0.78, and *I*^2^ = 0%) (Figure 4).

#### 3.4.2. Patients' Maximal Oxygen Consumption

In the age >50, the effect of sports on VO2 among kidney failure patients is insignificant (MD = −1.23, 95% CI [−2.75, 0.29], *P* = 0.11, *P* for heterogeneity = 0.15, and *I*^2^ = 40%); in the age between 40 and 50, exercise can also significantly reduce VO2 in patients with renal failure (MD = −1.56, 95% CI [−10.37, −1.78], *P* = 0.07, *P* for heterogeneity = 0.83, and *I*^2^ = 0%); in the age between 20 and 40, physical activity can significantly reduce VO2 in patients with renal failure (MD = −1.35, 95% CI [−2.24, −0.45], *P* = 0.003, *P* for heterogeneity = 0.44, and *I*^2^ = 0%) (Figure 5).

### 3.5. Sensitivity Analyses

To examine the stability of the outcome in blood pressure, a sensitivity analysis is needed. A relative outlier was excluded, and the result demonstrates that, in heterogeneity part, *I*^2^ changed from 77 to 2%. It indicates that the heterogeneity is mainly due to McMahon's report in 1999 (Figure 6).

### 3.6. Bias Analyses

A funnel plot for blood pressure and maximal oxygen consumption was performed. All the studies were included in the plot. To some extent, the result indicated that there existed some publication bias (Figure 7). The changes in the outcomes from baseline for blood pressure and VO2max were 11.6% and 88.4, respectively.

## 4. Discussion

Chronic renal failure is a severe clinical problem which has some significant socioeconomic impact worldwide. Despite advances in renal replacement therapies and organ transplantation, there exist abundant concerns like poor quality of life for dialysis patients and long transplantation waiting lists [14, 29, 30]. Besides the treatment to cure patients, the ways to improve the quality of patients' life are important. It is reported that the number of chronic kidney failures treated by hemodialysis is continuously increasing and most patients have reduced physical exercise and have a high risk of cardiac and vascular disease [31].

Physical activity program is suggested to help in making patients' life quality better. The activity is usually conducted mainly twice or three times per week, and the participation time is about 1 hour. The period ranges from 3 months to 1 year. The items of the exercise contain warm-up and strength and aerobic exercises. The studies about the necessity of physical activity showed that renal failure patients have seriously reduced physical capacity and they have a high risk of cardiac and vascular diseases. Therefore, physical exercise should be considered as both prevention and rehabilitation.

This meta-analysis aims to update and evaluate the effects of exercise on the health state in renal failure patients. The results in this study show that physical activity have benefits in blood pressure among sick people and improve their maximal oxygen consumption. These can help patients in physical function and aerobic capacity and may give them further benefits. These findings are in accord with the conclusion reported by Adams and Vaziri, which noted that exercise restores some level of physical performance and quality of life, which can be beneficial in patients with renal failure [15].

Our study also finds that the effects of exercise showed difference in various age groups. In the subgroup analyses of blood pressure, the elderly (age > 40) have significant improvement in controlling blood pressure, while young people' results (20 < age < 40) are insignificant. These may be because the condition of blood pressure in old people is worse compared to young man, and the change of blood pressure in old men is relatively easier to achieve. In the maximal oxygen consumption part, people in all the age ranges make their ability better after performing the exercise program. Jiang reported that diet and proper exercise were helpful in the elderly with chronic renal failure [32].

This meta-analysis includes the studies which are all from randomized trials. According to the GRADE quality-assessment scale, the quality of the individual studies in this meta-analysis was confirmed. To control selection bias, a sensitivity analysis was applied and found that McMahon's results were outliers and should be dropped. The result in this research is a suggestion both in scientific viewpoint and in clinical practice. However, there were some limitations in this article: the number of included researches was not abundant, and long-term effects of exercise on people with renal failure cannot be inferred in this study. Besides, methodological differences and confounding factors of selected studies were unavoidable.

## 5. Conclusion

Exercise program is associated with health state of people with kidney failure. Physical activity will improve body function and physical capacity, which will benefit patients with hemodialysis and help them in their blood pressure and maximal oxygen consumption. In spite of these benefits, the other potential effectiveness of exercise is needed. The results in the included randomized controlled trials could be more comprehensive. Besides, more randomized controlled trials are required to determine the influence of physical activity on a larger sampling size.

## Figures and Tables

**Figure 1:** Flow diagram of the study selection.

**Figure 2:** A forest plot for blood pressure of patients with chronic renal failure.

**Figure 3:** A forest plot for maximal oxygen consumption of patients with chronic renal failure.

**Figure 4:** A forest plot for the subgroup analyses of blood pressure in patients with chronic renal failure based on their age.

**Figure 5:** A forest plot for the subgroup analyses of maximal oxygen consumption in patients with chronic renal failure based on their age.

**Figure 6:** A forest plot of the subgroup analyses of blood pressure in patients with chronic renal failure for sensitivity test.

**Figure 7:** A funnel plot for blood pressure and maximal oxygen consumption in patients with chronic renal failure.

**Table 1:** Characteristics of RCT studies included in the meta-analysis.

Study	Year	Country	Period	Groups	Sampling Size	Age	Renal Failure Confirmation	Matching
Molsted et al.	2004	Denmark	1991–2000	Exercise	11	59	Medical records	Age, sex
				Control	9	48		
Henrique et al.	2010	Brazil	2003–2005	Exercise	7	47.6	Pathologically confirmed	Age
				Control	7	42.5		
Greenwood et al.	2015	UK	2010–2012	Exercise	8	53.8	Medical records	Age, sex
				Control	10	53.3		
Svarstad et al.	2002	Norway	1998–2000	Exercise	7	50	Medical records	Age
				Control	8	31		
Messonnier et al.	2012	France	2008–2010	Exercise	11	26.4	Pathologically confirmed	Age, sex
				Control	11	25.3		
McMahon et al.	1999	Australia	1996–1998	Exercise	5	58	Pathologically confirmed	Age, income
				Control	9	34		
Cupisti et al.	2004	Italy	1995–2002	Exercise	28	46	Medical records	Age, sex
				Control	28	43		
Cho and Sohng	2014	Korea	2000–2012	Exercise	23	60.8	Pathologically confirmed	Age, sex
				Control	23	57.7		
Li et al.	2012	China	1995–2011	Exercise	25	24.24	Medical records	Age
				Control	25	22.12		

## References

[1] Pinto A. R., da Silva N. C., Pinato L. (2016). Analyses of melatonin, cytokines, and sleep in chronic renal failure. *Sleep and Breathing*.

[2] Gündüz Z., Patiroglu T., Düsünsel R., Poyrazoglu M. H. (2001). 11-Year-old boy with chronic renal failure and myelodysplastic syndrome. *Pediatrics International*.

[3] Stiefelhagen P. (2002). Acute and chronic renal failure—prognosis depends on early diagnosis. *MMW—Fortschritte der Medizin*.

[4] Adnan T., Elif A. A., Ayşe K., Gülnaz A. (2005). Clonidine as an adjuvant for lidocaine in axillary brachial plexus block in patients with chronic renal failure. *Acta Anaesthesiologica Scandinavica*.

[5] Yilmaz M., Erol M. K., Cetinkaya R., Alp N. (2002). Effect of haemodialysis on left atrial mechanical function in patients with chronic renal failure. *Acta Cardiologica*.

[6] Liou H. H., Chiang S. S., Wu S. C., Yang W. C., Huang T. P. (1994). Intravenous infusion or nebulization of salbutamol for treatment of hyperkalemia in patients with chronic renal failure. *Zhonghua Yi Xue Za Zhi*.

[7] Chen S. F., Wang I. J., Lang H. C. (2016). Risk of major depression in patients with chronic renal failure on different treatment modalities: a matched-cohort and population-based study in Taiwan. *Hemodialysis International*.

[8] Kucur C., Ozbay I., Gulcan E., Kulekci S., Aksoy S., Oghan F. (2016). Evaluation of nasal mucociliary activity in patients with chronic renal failure. *European Archives of Oto-Rhino-Laryngology*.

[9] Su M.-S., Jiang Y., Yan X.-Y. H. (2013). Alcohol abuse-related severe acute pancreatitis with rhabdomyolysis complications. *Experimental and Therapeutic Medicine*.

[10] West H. (2007). Rhabdomyolysis associated with compartment syndrome resulting in acute renal failure. *European Journal of Emergency Medicine*.

[11] Wang T., Wu S. C., Yang W. C. (1995). Influence of peritoneal dialysis on the progression of chronic renal failure. *Advances in Peritoneal Dialysis*.

[12] Geary D. F., Ikse K. H., Coulter P., Secker D. (1990). The role of nutrition in neurologic health and development of infants with chronic renal failure. *Advances in Peritoneal Dialysis*.

[13] Flynn J. T., Frisch K., Kershaw D. B., Sedman A. B., Bunchman T. E. (1999). Response to early measles-mumps-rubella vaccination in infants with chronic renal failure and/or receiving peritoneal dialysis. *Advances in Peritoneal Dialysis*.

[14] Jungers P., Nguyen Khoa T., Joly D., Choukroun G., Witko-Sarsat V., Massy Z. A. (2000). Atherosclerotic complications in chronic renal failure: epidemiology and predictive factors. *Advances in Nephrology from the Necker Hospital*.

[15] Adams G. R., Vaziri N. D. (2006). Skeletal muscle dysfunction in chronic renal failure: effects of exercise. *American Journal of Physiology—Renal Physiology*.

[16] Salako B. L., Ayodele O. E., Kadiri S., Arije A. (2002). Prevalence of hepatitis B and C viruses in pre-dialysis patients with chronic renal failure. *African Journal of Medicine and Medical Sciences*.

[17] De Filippo M., Sverzellati N., Zompatori M. (2009). Unenhanced CT in patients with chronic renal failure with clinical suspicion of small-bowel infarct. *American Journal of Roentgenology*.

[18] Han S. Y., Witten D. M. (1977). Diffuse calcification of the breast in chronic renal failure. *American Journal of Roentgenology*.

[19] Molsted S., Eidemak I., Sorensen H. T., Kristensen J. H. (2004). Five months of physical exercise in hemodialysis patients: effects on aerobic capacity, physical function and self-rated health. *Nephron—Clinical Practice*.

[20] Messonnier L., Samb A., Tripette J. (2012). Moderate endurance exercise is not a risk for rhabdomyolysis or renal failure in sickle cell trait carriers. *Clinical Hemorheology and Microcirculation*.

[21] Henrique D. M. N., Reboredo M. D. M., Chaoubah A., De Paula R. B. (2010). Aerobic exercise improves physical capacity in patients under chronic hemodialysis. *Arquivos Brasileiros de Cardiologia*.

[22] Cho H., Sohng K.-Y. (2014). The effect of a virtual reality exercise program on physical fitness, body composition, and fatigue in hemodialysis patients. *Journal of Physical Therapy Science*.

[23] Cupisti A., Licitra R., Chisari C. (2004). Skeletal muscle and nutritional assessment in chronic renal failure patients on a protein-restricted diet. *Journal of Internal Medicine*.

[24] Greenwood S. A., Koufaki P., Mercer T. H. (2015). Effect of exercise training on estimated GFR, vascular health, and cardiorespiratory fitness in patients with CKD: a pilot randomized controlled trial. *American Journal of Kidney Diseases*.

[25] McMahon L. P., McKenna M. J., Sangkabutra T. (1999). Physical performance and associated electrolyte changes after haemoglobin normalization: a comparative study in haemodialysis patients. *Nephrology Dialysis Transplantation*.

[26] Svarstad E., Myking O., Ofstad J., Iversen B. M. (2002). Effect of light exercise on renal hemodynamics in patients with hypertension and chronic renal disease. *Scandinavian Journal of Urology and Nephrology*.

[27] Li Q. H., Wang S. M., Hu Z. X. (2012). Clinical analysis of 25 patients with secondary acute renal failure induced by rhabdomyolysis. *Chinese Journal of Integrated Traditional and Western Nephrology*.

[28] Worthley M. I., Unger S. A., Mathew T. H., Russ G. R., Horowitz J. D. (2003). Usefulness of tachycardic-stress perfusion imaging to predict coronary artery disease in high-risk patients with chronic renal failure. *The American Journal of Cardiology*.

[29] Ozdemir E., Koc Y., Kansu E. (2006). Successful treatment of chronic myeloid leukemia with imatinib mesylate in a patient with chronic renal failure on hemodialysis. *American Journal of Hematology*.

[30] Evans M., Fryzek J. P., Elinder C.-G. (2005). The natural history of chronic renal failure: results from an unselected, population-based, inception cohort in Sweden. *American Journal of Kidney Diseases*.

[31] De Vecchi A. F., Colucci P., Salerno F., Scalamogna A., Ponticelli C. (2002). Outcome of peritoneal dialysis in cirrhotic patients with chronic renal failure. *American Journal of Kidney Diseases*.

[32] Jiang H. (2013). Nursing experience of hemodialysis elder patients with renal failure. *Journal of Health*.

